# Prevalence of Asymptomatic Brucellosis in Children 7 to 12 Years Old

**DOI:** 10.1155/2015/187369

**Published:** 2015-10-20

**Authors:** Mohammad Aghaali, Siamak Mohebi, Hosein Heydari

**Affiliations:** ^1^Qom University of Medical Sciences, Qom 3713649373, Iran; ^2^Department of Public Health, Qom University of Medical Sciences, Qom 3713649373, Iran; ^3^Pediatric Medicine Research Center, Qom University of Medical Sciences, Qom 3713649373, Iran

## Abstract

*Background*. Brucellosis is one of the most common diseases of humans and animals and its clinical manifestations differ from asymptomatic infection to chronic illness associated with recurrence of symptoms. This study aimed to evaluate the prevalence of brucellosis in asymptomatic children 7 to 12 years old in Kahak, Iran. *Methods*. In this study, 186 children 7 to 12 years old were evaluated. Demographic data and exposure to the brucellosis agent were recorded and blood samples for the Wright, Coombs, and 2ME tests were collected. All the study subjects were followed up for one year about the appearance of symptoms. *Results*. The mean age was 10 ± 1.72 years and 51% were boys. Family history was positive for brucellosis in 15% of children. A total of 8 children were brucellosis seropositive and, in subsequent follow-up, 6 of them showed the disease symptoms. *Conclusion*. This study showed that approximately 4.3% of children in endemic areas can have asymptomatic brucellosis and many of these children may be symptomatic in short term.

## 1. Introduction

Brucellosis is a zoonosis disease caused by the bacterial genus* Brucella.* That is transmitted directly or indirectly by contact with infected animals or contaminated dairy products. Its clinical manifestations vary from asymptomatic infection to chronic forms.* Brucella* species are small, gram-negative, nonmotile, nonspore-forming, and rod-shaped (coccobacilli) bacterial organisms and 8 species of them have been identified. Four of them have moderate-to-significant human pathogenicity and include* Brucella abortus* (from cattle; moderate pathogenicity),* Brucella suis* (from pigs; high pathogenicity),* Brucella melitensis* (from sheep; highest pathogenicity), and* Brucella canis* [1, 2].

Typically, humans contract disease by ingesting contaminated food, such as unpasteurized milk products, but can also acquire it through inoculation via direct contact with infected animals or animal parts and occasionally through occupational exposure in microbiology laboratories [1]. Clinical classifications of brucellosis are subclinical, acute, subacute, chronic, and localized brucellosis. Brucellosis affects various organs and has nonspecific symptoms such as fever, bone and muscle pain, weakness, sweating, weight loss, and headache [1].

It is endemic in Iran and the most common agent is* Brucella melitensis* [3]. In endemic areas, a high percentage of patients with brucellosis are asymptomatic and less than 10% of them are diagnosed following infection in the early stages [4, 5]. Also in endemic areas, symptomatic patients only refer to health centers for diagnosis and treatment so asymptomatic patients remain carrier. These patients may present signs of infection in conditions such as reinfection or immune deficiency conditions [6].

In many countries, brucellosis is an occupational disease, which is uncommon in children. However, in Iran, because it is transmitted from animals to humans in nonoccupational ways, its prevalence in children is equal to adults or higher than them [7]. Clinical manifestations of brucellosis in children are like adults. However, being unfamiliar with the disease may be a delay in diagnosis [8]. By early diagnosis and effective treatment, many of these patients recover without any persistent complications. Given the high prevalence of brucellosis in Iranian children and the importance of diagnosing the asymptomatic patients, this study examined the prevalence of brucellosis in asymptomatic children 7 to 12 years old in Kahak, Iran.

## 2. Methods

This study was carried out at the first 6 months of 2013 in Kahak, Iran. The study population was all children aged 7 to 12 years. Children without a history of brucellosis and treatment for brucellosis and having typical signs of infection (fever, sweating, fatigue, and musculoskeletal pain) were included. Of 258 children, one hundred and eighty-six elementary school children met the inclusion criteria. A physician did history taking and physical examination for signs and symptoms of the disease. Children were enrolled after informing them and their parents of the study plan and obtaining informed consent from parents. All eligible study subjects consented to participate. The study was planned according to the ethical guidelines following the Declaration of Helsinki and Ethics Committee of Qom University of Medical Sciences approved it.

None of the study subjects had a history of vaccination against brucellosis. After selecting study subject, demographic data, history of exposure to the brucellosis agent, and type of the exposure were recorded. Then, 5 mL of venous blood was obtained for the Standard Tube Agglutination Test (STA: Wright) and Coombs and 2-Mercaptoethanol (2ME) tests. Tube agglutination testing was carried out using the Pasteur-protocol kit (Iranian Institute for Health Sciences Research Co., Tehran). To perform the Wright test, serum was diluted to 1/1280. Children with Wright test of ≥1/80 and 2ME ≥ 1/40 or Coombs Wright ≥ 1/80 were considered positive. All children were followed up for one year about the appearance of symptoms and were examined by the physician every two months. Study subjects were given notices to prevent the disease during the follow-up period. Data was analyzed using SPSS version 20 with Chi square and Fisher's exact test.

## 3. Results

A total of 186 children were enrolled. The mean age was 10 ± 1.72 years. Minimum and maximum ages of the study subject were 7 and 12 years, respectively. Subjects included 95 (51%) males and 91 (49%) females and 15% of them (28 cases) had family history of brucellosis. Animal contact was positive in 17.7% of children (33 cases) while 29% of them (54 cases) had a history of consumption of unpasteurized dairy products (Table 1).

At enrollment, Wright test was 1/160 in two children and 1/40 in two children and the rest of them had negative Wright test result. Positive Wright test children had 1/40 2ME result. Of the study subject who had negative Wright test, Coombs Wright test was 1/160 in 4 children, 1/80 in 2 children, and 1/40 in 20 children and it was negative in other study subjects. A total of eight children (3.4%) were seropositive (Wright test of ≥1/80 and 2-Mercaptoethanol (2ME) ≥ 1/40 or Coombs Wright ≥ 1/80).

All children were followed up for one year for the appearance of symptoms. Among eight seropositive study subjects, the symptoms manifested in six cases (Table 2).

These patients underwent standard treatment (Trimethoprim-sulfamethoxazole 10 mg/kg/day of Trimethoprim PO twice daily plus rifampin 15–20 mg/kg/day PO for 6 weeks). After 2 months of the treatment, 4 patients were 2ME negative (patients numbers 1, 2, 5, and 6; Table 2) and 2 patients had negative 2ME result after 4 months (patients numbers 3 and 4; Table 2) of treatment, and all clinical symptoms were resolved.

## 4. Discussion

Brucellosis is a zoonotic disease and, despite all efforts to reduce its incidence by vaccination of cattle and pasteurization of dairy products, it is still an important health problem in some parts of the world, especially in Asia and the Mediterranean [9, 10]. Its prevalence in Iran varies from 0.5 to 10.9% and its 5-year incidence rate in the central provinces of Iran is estimated to be 40–50 cases per 100,000 [11].

Previous studies have shown that zoonosis diseases may cause subclinical or asymptomatic infection in patients with persistent or occupational exposure to sources of the disease [12–14]. This could be due to frequent contact with the pathogen and a relative resistance to it. Identification and treatment of these patients is costly effective if its screening is economically cheaper than treating complications and treatment of patients in which the disease is transmitted by undiagnosed carriers [15].

This study aimed to evaluate the prevalence of asymptomatic brucellosis in children 7 to 12 years old in an endemic city. The results showed that, in endemic areas, asymptomatic brucellosis occurs in children with the incidence of 3.4%. Asymptomatic infection may result from contact with animals harboring low virulence species of* Brucella* or from less frequent contact with contaminated sources [6]. The importance of this issue is in the early detection, preventing chronic infection and finding the origin of the disease to prevent transmission to others. Zhen and colleagues showed that among 300 adults with continuous contact to animals and their products, 131 cases (45%) had asymptomatic brucellosis [6]. In another study by Çelebi et al., three members of a family with acute infection were studied by culture and all three members of the family (parents and sister of the patient) were infected with brucellosis. Also, the breast milk culture was positive for bacteria [16].

The most benefit of screening in endemic area is detection of new cases that are unaware of their disease because of lack of symptoms or mild symptoms such as fever and myalgia which did not require medical advice. These cases would not have been recognized without screening. However, early detection and prompt treatment of the disease can provide rapid recovery and prevent complications or sequels [17–19].

In Tabak's study, of 100 family members of patients with brucellosis, 20 cases were seropositive and, among them, 12 cases were asymptomatic and, within 6 to 12 months' follow-up, none of them had symptoms [20].

However, in the present study, 6 of 8 seropositive children became symptomatic during one year follow-up. Sofian et al. in a study evaluated 163 family members of 50 patients with acute brucellosis in an endemic area of Iran. 9.2% of family members were seropositive for* Brucella* agglutinin and, among them, 53.3% were asymptomatic and 46.7% were symptomatic. They showed that family members of brucellosis patients are at risk of disease acquisition, and screening of household members provides an effective way for early diagnosis and prompt treatment [3]. Almuneef et al. evaluated 404 household members of 55 patients with acute brucellosis in endemic areas of Saudi Arabia. Of the 404 household members screened, 53 were seropositive; of these 39 were symptomatic, and 9 had* Brucella* bacteraemia. They showed that screening family members of an index case of acute brucellosis would detect additional cases [21].

## 5. Conclusion

To our knowledge, this is the first study on the prevalence of brucellosis in asymptomatic children. It showed that, in endemic areas, about 4.3% of children may have asymptomatic brucellosis by which most of them may get symptomatic in short term. It seems that early detection can help timely treatment and prevention of the complications.

## Figures and Tables

**Table 1:** Distribution of risk factors for disease in children based on serological test result.

Risk factor	Seronegative (178)	Seropositive (8)	Total (186)	*P* value
Animal contact	27 (15.16%)	6 (75.0%)	33 (17.7%)	<0.001
Dairy consumption	46 (25.84%)	8 (100.0%)	54 (29.0%)	<0.001
Family history of brucellosis	24 (13.48)	4 (50.0%)	28 (15.0%)	0.005

**Table 2:** Epidemiological and clinical data of the 6 symptomatic children.

Patient	Age (years)	Gender	Symptoms during follow-up	Time of symptoms appearance (week)	Primary tests	Family history
1	8	Boy	Fever and sweating	8	Wright 1/160 and 2ME 1/40	+
2	7	Boy	Knee pain	30	Coombs Wright 1/160 and Wright negative	+
3	9	Boy	Abdominal and ankle pain	22	Coombs Wright 1/160 and Wright negative	−
4	8	Girl	Sacroiliitis	12	Coombs Wright 1/160 and Wright negative	−
5	10	Boy	Abdominal and knee pain	3	Coombs Wright 1/80 and Wright negative	+
6	10	Girl	Knee pain	8	Wright 1/160 and 2ME 1/40	−
